The article "Awareness of Gadolinium Toxicity Among Non-radiologists in Saudi Arabia" was published in 2022. Journal: Cureus.

# Awareness of Gadolinium Toxicity Among Non-radiologists in Saudi Arabia

**DOI:** 10.7759/cureus.21104

**Published:** 2022-01-11

**Authors:** Kholoud Sandougah, Raghad AlJohar, Dina Aladhadhi, Yara T AlHazmi, Marwh N Kariri, Khalid A Bin Abdulrahman

**Affiliations:** 1 Radiology, College of Medicine, Imam Mohammad Ibn Saud Islamic University, Riyadh, SAU; 2 Medicine, Imam Mohammed Ibn Saud Islamic University, Riyadh, SAU; 3 Medicine, Imam Mohammad Ibn Saud Islamic University, Riyadh, SAU; 4 Medicine, Imam Mohammed Ibn Saud Islamic University, Riyadh, Saudi Arabia, Riyadh, SAU; 5 Family and Community Medicine, Imam Mohammad Ibn Saud Islamic University, Riyadh, SAU

**Keywords:** renal toxicity, brain deposition, non-radiological doctor, enhanced mri, awareness, gadolinium

## Abstract

Introduction and aim

Gadolinium toxicity has been accompanied by side effects among patients scanned with MRI, especially patients with chronic renal insufficiency. The toxicity, pharmacokinetics, and pharmacodynamics of gadolinium-based contrast agents intact blood-brain barriers accumulate in the brain. This study aimed to estimate the awareness about the side effects of gadolinium-enhanced MRI scans among Saudi non-radiologists to improve and raise the level of awareness of all physicians about the side effects of gadolinium-enhanced MRI studies among patients. This improvement will be due to our clarification of the most important issues related to gadolinium contrast in MRI, by illustrating the uses and the major side effects of this contrast. Additionally, we want to find a method that will help with raising awareness of gadolinium toxicity and alert the stakeholders and the head of radiology departments about the need of creating and implementing new official regulations to minimize the abuse of enhanced MRI studies.

Materials and methods

This is a cross-sectional study conducted among non-radiological doctors in Saudi Arabia. A questionnaire based on a literature review was developed and distributed among non-radiological doctors through an online platform. The questionnaire included basic demographic data and a behavioral and awareness assessment about gadolinium. All statistical analyses were carried out using Statistical Package for the Social Sciences (SPSS) IBM Corp. Released 2019. IBM SPSS Statistics for Windows, Version 26.0. Armonk, NY: IBM Corp.

Results

460 non-radiological doctors contributed, 65% males vs. 35% females. The most commonly known side effect of gadolinium was acute pancreatitis (92.8%), followed by encephalopathy (90%) and arrythmias (88.9%). Awareness of gadolinium toxicity among the non-radiological doctors was poor in 74.6%, 20.9% were moderate, and only 4.6% were classified into a good awareness level. The factor associated with an increased level of awareness was being an internal medicine doctor (p=0.006).

Conclusion

The awareness level of non-radiological doctors about gadolinium toxicity was suboptimal. The knowledge of internal medicine physicians was better, but the other specialties need more education. As most of the physicians were not exposed to patients’ adverse reactions, this could be one of the reasons why they have a lack of knowledge about the subject. On the other hand, appropriate patient screening and sufficient prophylactic measures can prevent adverse events. Therefore, in knowledge, understanding, and practice, it is important to come up with the most effective response to any gadolinium contrast adverse events.

## Introduction

The first gadolinium chelates (GC) were used as contrast agents for magnetic resonance imaging (MRI) about 38 years ago [1]. Since its initial U.S. Food and Drug Administration (FDA) approval, gadolinium (Gd) has been widely used in clinical practice [2]. Gadolinium-based contrast agent (Gd) is one of the most widely recognized non-invasive methods used in patient clinical examinations in the world. Gd is considered toxic in the ionic state but relatively less toxic in the form of chelate [3]. However, the toxicity, pharmacokinetics, and pharmacodynamics of gadolinium-based contrasts (GBCs) have been examined with hawk eyes in recent reports that patients with normal kidney function will intact blood-brain barriers accumulate in the brain [4-7]. After repeated doses of contrast-enhanced magnetic resonance imaging, high signal intensity in the cerebellar structures was revealed [6]. Increased signal intensity in the dentate nucleus and globus pallidus on unenhanced T1-weighted images showed a positive correlation with previous exposure to linear chelate type gadolinium-based contrast agents, but not to macrocyclic chelate type gadolinium-based contrast agents (GBCAs), even in patients with normal renal function [7]. The stability of GBCAs is thought to be reflected in this discrepancy, and de-chelated gadolinium deposition has long been hypothesized [7]. Gadolinium was found in the brains of patients with a history of repeated GBCA administration using inductively coupled plasma mass spectrometry [7]. In certain situations, the gadolinium concentration in a patient's brain with the normal renal function was higher than the gadolinium concentration in the skin in individuals with nephrogenic systemic fibrosis, but there was no histological change [7]. Gadolinium is a lanthanide metal with paramagnetic properties, and this makes it a great IV material. The contrast (intra-blood vessel) strengthens the images of many tissues. Because it is a metal, it must be in an ionic form to be dissolvable in water and to be infused as a different profession; in any case, gadolinium in this free form [8]. Previous studies have shown that gadolinium is proportionally harmless when used in an appropriate clinical reference portion. However, unwanted symptoms may occur if there is an overdose or inappropriate use in some cases, and Gd chelates can cause intense renal disappointment in patients with chronic renal failure [9].

Most side effects of gadolinium are minor and have been classified into two groups: non-allergic reactions (e.g., headache, fatigue, arthralgia, loss of taste, flushed feeling, nausea, or vomiting) and other specific sensitivity responses, such as urticaria and diffuse erythema [10]. These patients are prone to nephrogenic systemic fibrosis [11-15]. Which mostly affects the skin, but may also include different organs, such as the muscle, liver, lungs, and heart; Gd particle MRI scans stimulate this disease since the half-life of these agents is extended 20 times past their normal half-life (about 90 minutes) [14,15]. Although the chelated form of less stable GCs has been proposed to play a role, the most commonly accepted hypothesis is the gradual release of dissociated gadolinium into the body, leading to systemic fibrosis. However, the entire chain of events is still not fully understood in a causal way, and many uncertainties remain [15]. Nephrogenic systemic fibrosis (NSF) is a scleroderma-like disease associated with the previous administration of gadolinium chelates. NSF occurs in patients with severe renal failure [15,16]. This disorder causes serious suffering, permanent disability, and increased mortality for those affected [17]. This correlation has led to guidance and best operational recommendations for use in renal insufficiency cases in public health counseling [16,17]. The lack of awareness about gadolinium toxicity, especially among non-radiological doctors in various fields, could therefore improve unwanted results in patients with gadolinium lethality. Our study aims to assess such awareness among non-radiologists in Saudi Arabia in general and in Riyadh in particular.

## Materials and methods

This was a cross-sectional study conducted among (n=450) non-radiological doctors in Saudi Arabia. A questionnaire is developed based on the literature review of topics related to gadolinium toxicity and side effects on patients and the awareness of the non-radiology physicians; it underwent a series of rehearsals and feedback. Final validation was performed with a group of non-radiology doctors who are not included in the final survey. Incorporation with Saudi Commission for Health Specialties, an email with an explanation and a link to the anonymous online survey (survey monkey forms) will be sent to non-radiology physicians in the Kingdom of Saudi Arabia (KSA). Then, they were reminded about the survey a week later. The questionnaire included basic demographic data and a behavioral and awareness assessment about gadolinium. All statistical analyses were carried out using Statistical Package for the Social Sciences (SPSS) IBM Corp. Released 2019. IBM SPSS Statistics for Windows, Version 26.0. Armonk, NY: IBM Corp.

Statistical analysis

Descriptive statistics were presented with numbers, percentages, mean, standard deviation, and median (IQR), whenever appropriate. The awareness of non-radiologists about gadolinium has been assessed using eight questions, where the correct answers have been identified and coded with one while the incorrect answers have been coded with 0. Items #3 and #8 (knowledge about gadolinium side effects) are multiple response answers. The total awareness was calculated by adding all eight items, and the total possible score range calculated was from 1-26 points, which generally means that the higher the score, the higher the awareness about gadolinium. Using 50% and 75% of the total score points to determine the level of awareness, patients were classified as having poor awareness if their score was less than 50% of the total score points, 50%-75% were classified as having moderate awareness, and above 75% of the total score points were classified as a good awareness level. The awareness scores were compared to the sociodemographic characteristics of the patients by using the Mann-Whitney U test and Kruskal-Wallis test as applied. Normality tests were conducted using Shapiro-Wilk, Kolmogorov, and Smirnov tests. Data followed abnormal distribution. Thus, non-parametric tests were applied. Two-tailed analysis with p < 0.05 was used as the cutoff for statistical significance. All data analyses were performed using Statistical Package for the Social Sciences, version 26 (SPSS, Armonk, NY: IBM Corp, USA)

## Results

In this study, we recruited 460 non-radiologists to measure their awareness regarding gadolinium toxicity. Table 1 presents the basic demographic characteristics of the respondents. Nearly two-third (65%) were males, with approximately one-third (32.6%) being consultants and 29.3% residents. The most common specialty was a general practitioner (19.8%), followed by the surgeon (19.3%) and internal medicine (18.5%).

**Table 1:** Basic demographic data of the non-radiological doctors (n=460)

Study Data	N (%)
Gender	
Male	299 (65%)
Female	161 (35%)
Clinical classification	
General physician	97 (21.1%)
Resident	135 (29.3%)
Registrar	78 (17%)
Consultant	150 (32.6%)
Specialty	
Internal medicine	85 (18.5%)
Surgeon	89 (19.3%)
Family physician	55 (12%)
Ob-Gyne	27 (6%)
Pediatrician	37 (8%)
General practitioner	91 (19.8%)
Oncologist	12 (2.6%)
Others	64 (13.9%)

The behavior of the non-radiological doctors toward enhanced MRI and its side effects among patients is represented in Table 2. It can be observed that 43.9% of physicians would order an enhanced MRI in about one to two out of five cases. The proportion of physicians who reported that their patients experienced side effects after undergoing enhanced MRI was 8.5%, and the most commonly reported side effect was allergy (32.1%). Furthermore, the most commonly mentioned method to raise awareness of gadolinium was “a systematic auto-notification letter that appears upon requesting an MRI with contrast” and “an official controlling policy raised by radiology department to minimize the gadolinium-enhanced procedure” (37.4%).

**Table 2:** Non-radiological doctors’ behaviors toward enhanced MRI contrast and its side effects among patients (n=460) * Variable with multiple responses

Variables	N (%)
For every 5 cases, in how many cases do you order an enhanced MRI study?	
1 – 2 cases out of 5	202 (44%)
2 – 3 cases out of 5	57 (12.4%)
3 – 4 cases out of 5	33 (7.2%)
4 – 5 cases out of 5	19 (4%)
Never ordered a contrast enhanced study	149 (32.4%)
Did any of your patients experience side effects post-MRI study with contrast?	
Yes	39 (08.5%)
No	274 (59.6%)
I don’t know	147 (32%)
Side effect of gadolinium among patients^(n=28)^	
Allergy	09 (32%)
Nausea and vomiting	06 (21.4%)
Renal failure	06 (21.4%)
Other	07 (25%)
In your opinion, what are the effective ways to raise awareness about gadolinium-enhanced MRI (gadolinium agent, types, indications, and side effects)?*	
Hard copy memorandum to the head of departments	77 (16.7%)
Electronic memorandum to the head of departments	105 (22.8%)
A systematic auto-notification letter that appears upon requesting an MRI with contrast	272 (59%)
An official controlling policy raised by radiology departments to minimize the gadolinium-enhanced procedure	172 (37.4%)

The assessment of awareness about gadolinium toxicity among non-radiological doctors is described in Table 3. It was shown that 44.1% of the physicians were aware of the name, type, and chemistry of the contrast material used in MRI. Of these, 39.1% regularly consulted a radiologist before ordering a contrast-enhanced MRI study. When asked what needed to be checked in the patients before ordering an enhanced MRI study, based on multiple response answers, creatinine level (78.9%), previous side effects (70.2%), and any attached metallic objects (64.3%) were the top three most commonly stated factors. The proportion of physicians who believed that gadolinium is safe was 18.9%, while the proportion of physicians who had prior knowledge about NSF was 43.3%. Those physicians with prior knowledge about gadolinium brain deposition constituted 23%. Furthermore, 58% of the physicians strongly agreed that all practicing physicians should have prior knowledge about contrast materials and their side effects.

**Table 3:** Assessment of the non-radiologists’ awareness about Gadolinium toxicity (n=460) † Indicates correct answer, * Variable with multiple responses.

Statement	N (%)
Do you know the name, type, and chemistry of the contrast material used in MRI studies?	
Yes ^†^	203 (44%)
No	154 (33.5%)
I don’t know	103 (22.4%)
Do you consult a radiologist before ordering a contrast-enhanced MRI study?	
Yes ^†^	180 (39%)
No	158 (34.3%)
Occasionally	122 (26.5%)
3. From your experience, patients going through MRI with contrast study should be checked for: *	
Previous side effects ^†^	323 (70.2%)
Creatinine level ^†^	363 (79%)
Pregnancy ^†^	285 (62%)
Hormone therapy and other medications ^†^	100 (21.7%)
Any attached metallic objects ^†^	296 (64.3%)
Epilepsy ^†^	146 (31.7%)
I am not sure	45 (09.8%)
Others	25 (05.4%)
Do you think that gadolinium (the MRI contrast material) is safe?	
Yes	87 (19%)
It has minimal (treatable) side effects	173 (37.6%)
No ^†^	59 (12.8%)
I don’t know	141 (30.7%)
5. Do you have prior knowledge about nephrogenic systemic fibrosis (NSF)?	
Yes ^†^	199 (43.3%)
No	163 (35.4%)
I don’t know	98 (21.3%)
Do you have prior knowledge about gadolinium brain deposition?	
Yes ^†^	106 (23%)
No	246 (53.5%)
I don’t know	108 (23.5%)
Do you agree that all practicing physicians should have proper knowledge about contrast materials and their side effects?	
Strongly disagree	01 (0.2%)
Disagree	11 (2.4%)
Neutral	41 (9%)
Agree	140 (30.4%)
Strongly agree ^†^	267 (58%)
Total Awareness Score	
Mean ± SD	9.51 ± 5.16
Median (IQR)	9.00 (7.00)

In addition, in Figure 1, the most common side effects indicated by the physicians were acute pancreatitis (92.8%), encephalopathy (90%), arrhythmias (88.3%), paresthesia (86.3%), tachycardia (83.3%) and facial edema (81.5%) while the least of them was nausea (52.6%). Based on the above eight-item awareness questionnaires, the overall mean score was 9.51 ± 5.16.

**Figure 1:** Knowledge about the side effects of gadolinium † In Figure 1, the most common side effects indicated by the physicians were acute pancreatitis (92.8%), encephalopathy (90%), arrhythmias (88.3%), paresthesia (86.3%), tachycardia (83.3%), and facial edema (81.5%), while the least was nausea (52.6%). Based on the above eight-item awareness questionnaire, the overall mean score was 9.51 ± 5.16.

Figure 2 shows the level of awareness toward gadolinium toxicity. It was revealed that nearly three quarters (74.6%) were classified into poor awareness, 20.9% were moderate and the rest were poor (4.6%). 

**Figure 2:** Level of awareness about Gadolinium toxicity Shows the levels of awareness about gadolinium toxicity. It was revealed that nearly three-quarters (74.6%) were classified into poor awareness, 20.9% were moderate, and the rest were good (4.6%).

When measuring the differences in the awareness scores of the physicians in relation to the basic demographic data, it was found that the median score of internal medicine physicians was statistically significantly higher than the other groups of physicians (H=19.807; p=0.006) while the awareness scores of gender (U=23180; p=0.512) and position (H=4.282; p=0.233) were not significantly different across the groups (Table 4). 

**Table 4:** Difference in the awareness scores of non-radiological doctors (n=460) a P-value has been calculated using the Mann-Whitney U-test, b P-value has been calculated using the Kruskal-Wallis test, ** Significant at p<0.05 level.

Factor	Awareness Total score (26) Median (IQR)	U/H-test	P-value ^§^
Gender			
Male	9.00 (8.00)	U=23180	0.512
Female	9.00 (7.00)		
Clinical classification			
General physician	8.00 (7.00)	H=4.282	0.233
Resident	9.00 (6.00)		
Registrar	8.00 (7.00)		
Consultant	9.00 (8.00)		
Specialty			
Internal medicine	11.00 (9.00)	H=19.807	0.006 **
Surgeon	10.00 (9.00)		
Family physician	07.00 (7.00)		
Ob-Gyne	07.00 (4.00)		
Pediatrician	08.00 (5.00)		
General practitioner	09.00 (5.00)		
Oncologist	10.50 (5.50)		
Others	09.00 (7.50)		

## Discussion

This study attempted to evaluate the awareness of non-radiological doctors about gadolinium toxicity. The findings of this study showed that most of the non-radiological doctors had insufficient awareness about gadolinium toxicity: 74.6% of them were classified into the poor level, 21% were moderate, and only 4.6% were at a good awareness level (mean score: 9.51 out of 26 points). We also noted that internal medicine physicians had significantly better awareness scores, while family and ob-gyn physicians exhibited significantly lower awareness scores than the others (p=0.006). There have been limited studies that measure the overall awareness of physicians about enhanced MRI contrast. However, a study published in Malaysia evaluated radiographers’ knowledge regarding contrast media used in radiological procedures [18]. The findings revealed that radiographer knowledge about contrast media was moderate (77.8%). They further recorded that radiographers working for more than 10 years had better knowledge of contrast media than radiographers with less than 10 years of service. It is predicted that radiographers’ knowledge about contrast media is higher than that of physicians, as one may argue that the practice of the radiographer is different from the practice of the physician. In North America [19], investigators reported that radiologists were more aware of brain gadolinium depositions than non-radiologist physicians, and they were significantly more comfortable addressing patients’ inquiries than referring pediatric physicians. In our study, only 23% of the non-radiological doctors were aware of gadolinium brain deposition. In the USA [20], researchers reported that neurosurgeons and neuro endocrinologists were sometimes unaware of which contrast agents are used by their institutions, and many were also unaware that evidence of long-term brain retention has been reported with the use of gadolinium-based contract agents (GBCAs) in patients with normal functions. Furthermore, they reported that a lack of prior knowledge of new possible retention concerns regarding gadolinium in patients with normal renal function was reported by 28%, which was in line with our results.

On further assessment of awareness about gadolinium toxicity, we noticed that a little below half of the respondents (44.1%) knew the name, type, and chemistry of the contrast material used in MRI studies, and 39% of them regularly consulted radiologists to determine whether contrast-enhanced MRI is needed. On the other hand, physicians showed better knowledge that creatinine levels (78.9%), previous side effects (70.2%), any attached metallic objects (64.3%), and pregnancy (62.0%) should be checked among patients before undergoing MRI contrast. However, few of them (12.8%) thought that MRI contrast material was not safe. Despite this, most (58%) still strongly agreed that all practicing physicians should have proper knowledge about contrast materials and their adverse effects. A study by Beckett et al. [21]. documented that radiologists were not confident in handling adverse incidents, particularly the rare severe reactions due to contrast media, and they concluded that proper patient screening and adequate prophylactic measures can prevent some adverse reactions.

Moreover, nearly half of the physicians (43.3%) were knowledgeable about NSF. Knowledge about nephrogenic systemic firbrosis (NSF) among physicians is equally important since NSF occurs after receiving GBCA, and patients who have severe chronic or acute renal failure could be at higher risk of having an adverse reaction [21]. Studies suggest that NSF mainly affects the skin but may also affect other organs, such as the lungs, pleura, skeletal muscle, heart, and kidneys [22]. As Schlaudecker and Bernheisel reported, due to the large number of patients with clinically silent renal impairment and the serious consequences of NSF related to gadolinium exposure, physicians should use alternative imaging modalities for patients who are at risk [23]. It can be further observed that according to the knowledge of physicians, the most common side effect of gadolinium was acute pancreatitis (92.8%), followed by encephalopathy (90%), arrhythmias (88.9%), paresthesia (86.3%), and tachycardia (83.3%), while nausea (52.6%) was the least mentioned by the physicians as a side effect of enhanced gadolinium. Beckett et al. [21]. indicated that the most common adverse effect after going through enhanced contrast media was allergy. They further explained that although minor allergies are common to this method and do not pose an increased overall risk, a history of severe atopy, such as multiple allergies, or a prior major anaphylactic response, should heighten concern before ordering contrast media.

As for physicians’ behavior toward enhanced MRI, the data in this study revealed that 43.9% of the physicians ordered enhanced MRI in one to two cases out of five, but 32.4% had never ordered this method. In addition, the adverse events reported by their patients were low (8.5%), and allergy was the most commonly side effects] among patients. Physicians believed that the most effective way to raise awareness about gadolinium, including gadolinium agent, types, indications, and side effects, was through a systematic auto-notification letter appearing upon requesting an MRI with contrast (59.1%). 

## Conclusions

The awareness level of non-radiological doctors about gadolinium toxicity was suboptimal. The knowledge of internal medicine physicians was better, but the other specialties need more education. As most of the physicians were not exposed to patients’ adverse reactions, this could be one of the reasons why they have a lack of knowledge about the subject. On the other hand, appropriate patient screening and sufficient prophylactic measures can prevent adverse events. Therefore, in knowledge, understanding, and practice, it is important to come up with the most effective response to any gadolinium contrast adverse events. That could be achieved by adding gadolinium toxicity as a considerable objective in students' radiology curriculum than a further course for non-radiologists board doctors about contrast materials under the supervision of patients safety unit in the hospital. Furthermore, a systematic auto-notification letter that appears when requesting an MRI with contrast to the covering physician, and an official controlling policy raised by the radiology department would effectively minimize the gadolinium-enhanced operation. In addition to primary awareness by the ministry of health to the patients and the community.
